The article "Broadband Design of Midinfrared Chiral Metamaterials Based on the Indium Tin Oxide Conical Helix" was retracted in 2023. Reasons: signs of a paper mill; suspected computer-generated content; unreliable results or conclusions; concerns about the data.

# Broadband Design of Midinfrared Chiral Metamaterials Based on the Indium Tin Oxide Conical Helix

**DOI:** 10.1155/2022/3644004

**Published:** 2022-06-22

**Authors:** Wenmei Zhang

**Affiliations:** Xuzhou Technician College, Xuzhou, Jiangsu 221140, China

## Abstract

This paper proposed a periodic midinfrared broadband chiral structure composed of indium tin oxide (ITO) conical helix. The simulation results show that the structure achieves a good broadband CD in the midinfrared. At the wavelength of 9.2 *μ*m, the maximum value of CD is 0.55, the FWHM (full width half maximum) of CD is 7.2 *μ*m, and the wavelength range is from 5.7 *μ*m to 12.9 *μ*m. The simulation results also show that compared with the traditional uniform spiral structure with the same radius, the conical spiral structure can achieve better broadband circular dichroism in the midinfrared band. This provides a new idea for the design of broadband polarization state control devices in the midinfrared band.

## 1. Introduction

A midinfrared laser has important applications in communication, medical treatment, national defense, and so on. The effective control of midinfrared laser transmission is an important factor to determine whether the midinfrared laser can be better applied. The regulation of the midinfrared laser polarization state is the key link in midinfrared laser transmission control. As a new type of artificial electromagnetic material, chiral metamaterials have been widely studied and show strong ability in polarization state regulation [1–5]. Chiral metamaterials introduce chiral structures into metamaterials. It has two important properties [6]. Since the chiral properties of chiral metamaterials only occur near the oscillation wavelength of the structure, the reported response wavelengths of chiral metamaterials are mainly distributed in microwave [7], terahertz [8], visible light, or near-infrared region [9–17], and a small number of documents [18–21] report that the response wavelengths are distributed in the midinfrared band. For the study of circular dichroism, on the one hand, people seek a strong CD response. Because the CD response depends on the unit structure size and periodic array arrangement of chiral metamaterials, the bandwidth of this kind of research is mostly limited to a narrow wavelength range [22–26]. How to expand the bandwidth of CD response has become another research direction of circular dichroism [18, 27–29]. And chiral metamaterials mainly use traditional metal materials such as copper, silver, and gold. These metals have many shortcomings [30]. These deficiencies will affect the bias state regulation characteristics of chiral metamaterials in the midinfrared band composed of traditional metals. In view of the shortcomings of traditional metal materials, researchers have been looking for better plasmon materials in the midinfrared band. Metal oxide [30] shows metal characteristics in the midinfrared region. It has the advantages of the low real part of dielectric constant and good chemical stability. It can replace traditional plasmon materials such as gold and silver. In this paper, indium tin oxide (ITO) is selected as the plasmon material and designed into a conical spiral structure.

The article "Broadband Design of Midinfrared Chiral Metamaterials Based on the Indium Tin Oxide Conical Helix" was retracted in 2023. Reasons: signs of a paper mill; suspected computer-generated content; unreliable results or conclusions; concerns about the data.

## 2. Structure and Simulation

As shown in Figure 1, the metamaterial designed in this paper is a periodic array structure. Each cycle consists of a conical spiral, that is, the radii of the upper and lower ends of the spiral are different. The constituent material of the helix is ITO, and the base material is silicon. The radius of the conical spiral gradually increases from top to bottom. The radius of the upper end is *R*1 = 0.4 *μ*m, the radius of the lower end is *R*2 = 0.8 *μ*m, the radius of the spiral line is *r* = 0.2 *μ*m, the pitch is *p* = 2 *μ*m, the number of spiral turns is *n* = 3, and the cycle is *a* = 2.4 *μ*m.

FDTD software is used for simulation. Due to the periodicity of the structure, a unit is selected for simulation. It is assumed that right-handed circularly polarized light (RCP) and left-handed circularly polarized light (LCP) are incident along the positive direction of the *Z* axis, respectively. The two boundaries in the *Z* direction are set as perfectly matched layer (PLMS) boundary conditions. The boundaries in the *X* and Y directions are set as periodic boundary conditions. The dielectric constant of a Si substrate comes from experimental data [31], and the dielectric constant of ITO adopts the Drude–Lorentz model [30].

## 3. Simulation Results and Discussion

### 3.1. Principle Analysis

Through FDTD simulation, the transmission spectra of RCP light and LCP light calculated, respectively, are substituted into the following circular dichroism CD formula:

(1) $$\begin{array}{c} C\;D=\left|T_{+}-T_{-}\right|. \end{array}$$

The CD spectrum with the wavelength in the range of 4–14 *μ*m can be obtained, as shown in Figure 2, where *T*_+_ and *T*_−_ represent the light transmittance of RCP and LCP, respectively. It can be seen from the figure that in this band range, there is an obvious difference in the transmittance between right-handed circularly polarized light and left-handed circularly polarized light, resulting in obvious CD characteristics of the structure. Assuming that the FWHM (full width half maximum) of CD is the coverage of the wavelength when the maximum value of CD decreases to half. The CD FWHM of the structure is 7.2 *μ*m, and the wavelength range is from 5.7 *μ*m to 12.9 *μ*m. In the wavelength range of 4.5–14 *μ*m, the transmittance of LCP light is greater than that of RCP light. The reason is that the model selected in this paper is a right-handed spiral structure. When the RCP light is incident, the circular polarization direction of the electromagnetic wave is the same as the rotation direction of a spiral structure. Strong plasmon oscillation occurs in ITO, and the plasmon material constituting the spiral structure and the oscillation absorption is enhanced. When the LCP light is incident, the circular polarization direction of the electromagnetic wave is opposite to the rotation direction of the spiral structure. The plasmon oscillation in ITO is weaker, and the absorption is weaker than that in right-handed circular polarization. Thus, the transmittance of the LCP light is greater than that of the RCP light, resulting in obvious CD phenomenon. This result can also be proved from the absorption spectra of the RCP light and LCP light by the conical helix in Figure 3. It can be seen from Figure 3 that the transmittance of the LCP light is greater than that of the RCP light in the range of wavelength 4.6–14 *μ*m.

The article "Broadband Design of Midinfrared Chiral Metamaterials Based on the Indium Tin Oxide Conical Helix" was retracted in 2023. Reasons: signs of a paper mill; suspected computer-generated content; unreliable results or conclusions; concerns about the data.

### 3.2. Parameter Discussion

#### 3.2.1. Variation of the Radius Ratio

In this paper, the conical helix with a helix radius of 0.8 *μ*m from the base is selected, which is successively reduced upward to a helix radius of 0.4 *μ*m. We define the ratio of the lower spiral radius to the upper spiral radius as the radius ratio. The CD characteristics of the conical helix with a radius ratio of 1, 1.5, and 2 are simulated, respectively, as shown in Figure 4 where the radius ratio of 2 is the conical spiral structure as previously discussed, while the radius ratio of 1 is the uniform spiral structure with a constant radius. It can be seen from the figure that with the increase in the radius ratio, the response wavelength of CD changes red. Moreover, the broadband range is also significantly increased. The carriers in chiral metamaterials form plasmon oscillations under the action of an external electromagnetic field. The nature of the oscillations is related to the size of the structure. As can be seen from Figure 4, as the radius ratio gradually increases, the size of the maximum helix radius contained in the structure increases. The position of plasmon oscillation moves towards the long wavelength direction, so the peak value of CD appears to be a red shift. As for the bandwidth of CD, with the increase in the radius ratio, the range of spiral radius contained in the same spiral structure increases and the bandwidth of CD widens, which provides a design idea for obtaining broadband CD.

The article "Broadband Design of Midinfrared Chiral Metamaterials Based on the Indium Tin Oxide Conical Helix" was retracted in 2023. Reasons: signs of a paper mill; suspected computer-generated content; unreliable results or conclusions; concerns about the data.

#### 3.2.2. Variation of the Helix Radius

The helix radius in the structure is changed as shown in Figure 1, and the helix radius is taken 0.15 *μ*m, 0.20 *μ* m, and 0.25 *μ*m, respectively. Other parameters remain unchanged. The CD simulation results of the structure are shown in Figure 5. At the same time, with the increase in the helix radius, the size of the structure increases accordingly, the oscillation wavelength range of the structure also increases, and the bandwidth increases.

#### 3.2.3. Change in the Number of Spiral Turns

The number of turns of the spiral in the structure is changed as shown in Figures 1–4 turns, respectively, and other structural parameters remain unchanged. Their CDs are simulated, respectively, and the results are shown in Figure 6. The figure shows that with the increase in the number of turns, the peak value of CD moves to the long-wavelength direction, and the CD value changes slightly. The CD of the conical spiral with the number of turns of 3 has the maximum value.

## 4. Conclusion

In order to overcome the shortcomings of traditional midinfrared laser polarization state regulation, such as large volume, high cost, and difficult integration, in this paper, a chiral metamaterial in the midinfrared band is designed. The midinfrared plasmon material, ITO, is introduced into the chiral superstructure. A conical helical periodic chiral structure with ITO as the plasmon material is proposed, and the broadband CD in the midinfrared band is realized. In this paper, the CD characteristics of the structure in the 4 to 14 *μ*m band are simulated and calculated. At the wavelength of 9.2 *μ*m, the maximum value of CD is 0.55 and the FWHM of CD is 7.2 *μ*M. The simulation results show that the bandwidth of CD can be widened by increasing the radius ratio. Compared with the uniform spiral structure with the same radius, the conical spiral has more advantages in realizing the broadband of CD. This paper also discusses the influence of the number of turns of the conical helix and the radius of the helix on the CD structure.

## Figures and Tables

**Figure 1:** The schematic diagram of a chiral unit cell composed of a tapered helix.

**Figure 2:** CD and transmittances of the structure for the RCP and LCP incident waves.

**Figure 3:** Absorption spectra of the structure for the RCP and LCP incident waves.

**Figure 4:** CD properties of the structure with the different radius ratios of 1.0, 1.5, and 2.0, respectively.

**Figure 5:** CD properties of the structures with the different wire radii of 0.15 *μ*m, 0.20 *μ*m, and 0.25 *μ*m, respectively.

The article "Broadband Design of Midinfrared Chiral Metamaterials Based on the Indium Tin Oxide Conical Helix" was retracted in 2023. Reasons: signs of a paper mill; suspected computer-generated content; unreliable results or conclusions; concerns about the data.

**Figure 6:** CD properties of the structure with the different number of turns of the helix, 2 turns, 3 turns, and 4 turns, respectively.

## Data Availability

The data used to support the findings of this study are available from the author upon request.
